RETRACTED

# Receptor tyrosine kinase inhibitor Sunitinib and integrin antagonist peptide HM-3 show similar lipid raft dependent biphasic regulation of tumor angiogenesis and metastasis

**DOI:** 10.1186/s13046-019-1324-7

**Published:** 2019-08-28

**Authors:** Jialiang Hu, Wenjing Wang, Chen Liu, Mengwei Li, Edouard Nice, Hanmei Xu

**Affiliations:** 1 State Key Laboratory of Natural Medicines, Ministry of Education, China Pharmaceutical University, Nanjing, 210009 People’s Republic of China; 2 The Engineering Research Center of Synthetic Polypeptide Drug Discovery and Evaluation of Jiangsu Province, Nanjing, 211198 People’s Republic of China; 3 Department of Biochemistry and Molecular Biology, Monash University, Clayton, VIC 3800 Australia

**Keywords:** Tumor metastasis, Angiogenesis, Integrins, Cell migration, RhoGTPase, Lipid rafts

## Abstract

**Background:**

Anti-angiogenesis remains an attractive strategy for cancer therapy. Some anti-angiogenic reagents have bell-shape dose-response curves with higher than the effective doses yielding lower anti-angiogenic effects. In this study, two different types of anti-angiogenic reagents, a receptor tyrosine kinase inhibitor Sunitinib and an integrin antagonist peptide HM-3, were selected and their effects on tumor angiogenesis and metastasis were compared. The involved molecular mechanisms were investigated.

**Methods:**

The effect of high dose Sunitinib and HM-3 on tumor angiogenesis and metastasis was investigated with two animal models: metastasis of B16F10 cells in syngeneic mice and metastasis of human MDA-MB-231 cells in nude mice. Furthermore, mechanistic studies were performed with cell migration and invasion assays and with biochemical pull-down assays of intracellular RhoGTPases. Distribution of integrin αvβ3, α5β1, VEGFR2 and the complex of integrin αvβ3 and VEGFR2 inside or outside of lipid rafts was detected with lipid raft isolation and Western-blot analysis.

**Results:**

Both Sunitinib and HM-3 showed a bell-shape dose-response curve on tumor angiogenesis and metastasis in both animal models. The effects of Sunitinib and HM-3 on endothelial cell and tumor cell proliferation and migration were characterized. Activation of intracellular RhoGTPases and actin stress fiber formation in endothelial and cancer cells following Sunitinib and HM-3 treatment correlated with cell migration analysis. Mechanistic studies confirmed that HM-3 and Sunitinib regulated distribution of integrin αvβ3, α5β1, VEGFR2 and αvβ3-VEGFR2 complexes, both inside and outside of the lipid raft regions to regulate endothelial cell migration and intracellular RhoGTPase activities.

**Conclusions:**

These data confirmed that a general non-linear dose-effect relationship for these anti-angiogenic drugs exists and their mechanisms are correlative. It also suggests that the effective dose of an anti-angiogenic drug may have to be strictly defined to achieve its optimal clinical effects.

RETRACTED

**Electronic supplementary material:**

The online version of this article (10.1186/s13046-019-1324-7) contains supplementary material, which is available to authorized users.

## Background

Anti-angiogenesis is an attractive strategy for cancer therapy [1]. Sunitinib is a second-generation tyrosine kinase inhibitor that targets multiple tyrosine kinases, including the vascular endothelial growth factor receptors (VEGFRs), which play a role in both tumor angiogenesis and tumor cell proliferation.

Sunitinib has been validated for the treatment of renal cell carcinoma and gastrointestinal stromal tumor [2, 3]. However, recent specific examples have indicated that VEGF-targeted drugs inhibited primary tumor growth but ultimately shortened survival of mice by promoting tumor invasiveness and metastasis [4, 5]. Several plausible mechanisms were proposed including pruning quiescent vessels in healthy tissues to promote seeding of metastasizing tumor cells, or inducing a chronic “inflamed” state characterized by elevated levels of cytokines that stimulate metastasis and angiogenesis [6–8]. Interestingly, the dose of Sunitinib used (120 mg/kg/d) was higher than its effective dose in inhibiting primary tumor growth (60 mg/kg/d) [9]. Therefore, careful studies of the dose-response effects of Sunitinib are required to better understand its mechanism of action.

Some integrin antagonists also display anti-angiogenic activity [10]. An integrin antagonist peptide HM-3 with both anti-angiogenic and anti-tumor activity has recently entered clinical trials in China. Peptide HM-3 was constructed by connection of RGD to the C terminus of the ES-2 peptide with a glycine linker [11]. RGD is a tri-peptide sequence that has a high affinity to integrin αvβ3. ES-2, corresponding to amino acids 60–70 of endostatin, inhibits endothelial cell migration and differentiation by binding to integrin α5β1 [11, 12]. Interestingly, at a concentration of 4.5 μM, HM-3 inhibited endothelial cell (EAhy926) migration but promoted it at 17.8 μM [13]. Likewise, HM-3 at 3 mg/kg/d inhibited the growth of hepatic carcinoma SMMC-7721 in nude mice whereas at 48 mg/kg/d, it promoted this process in the same model [13].

In the current study, in vivo metastasis models were used in mice to confirm that these different anti-angiogenic reagents had a similar and non-linear dose-response relationship in the regulation of tumor metastasis and angiogenesis. In vitro cell migration assays and intracellular RhoGTPase activity assays were used for cellular studies. Importantly, RhoGTPases are central regulators of cell migration [14–17]. As HM-3 regulated EAhy926 cell migration in a glypican-1-dependent manner and glypican-1 only exists in the lipid raft region, we extended the study to distribution analysis of integrins (targets of HM-3) and VEGFR2 (a target of Sunitinib) inside or outside of lipid raft regions.

RETRACTED

Lipid rafts are specialized membrane microdomains to which transmembrane proteins and intracellular signaling molecules are recruited [18] (e.g. glycosylphosphatidylinositol (GPI)-anchored proteins and Src family kinases [19, 20]). Integrins αvβ3 and α5β1 can also be recruited into lipid rafts where they interact with local kinases and phosphatases to promote downstream signaling [21]. These integrins are recruited into lipid rafts via simultaneous interactions of their ligands (e.g. HM-3) with glypican-1, a sulfate proteoglycan that only exists in lipid rafts but does not have a signaling function per se [12]. Integrins in lipid rafts activate the FAK/Src (Focal Adhesion Kinase/Src family kinase) intracellular complex, which regulates the activities of Rac1 and RhoA via various guanine nucleotide exchange factors (GEFs) or GTPase-activating proteins (GAPs) and subsequently regulates the actin cytoskeleton. Such mechanisms of regulation ultimately lead to changes in cell migration [22].

Regulation of endothelial cell migration by integrins and VEGFR2 are not independent events [23]. Physical interactions and cross activation of integrin αvβ3 and VEGFR2 have been reported [24]. By their mechanistic study, Mahabeleshwar et al. found that VEGFR2 activation induced c-Src dependent β3 integrin tyrosine phosphorylation, which in turn is crucial for VEGF-induced tyrosine phosphorylation of VEGFR2 [25]. This provides insights into how integrin αvβ3 and VEGFR2 may promote HUVEC migration.

The Rho family GTPase Cdc42, Rac1 and RhoA regulate the actin cytoskeleton when cells are triggered via growth factor receptors and integrins [26, 27]. Rac1 and Cdc42 stimulate the formation of protrusive structures such as membrane ruffles, lamellipodia and filopodia. RhoA regulates contractility and assembly of actin stress fibers and focal adhesions [14]. Our data show that the signal transduction pathways of HM-3 and Sunitinib converge at the levels of intracellular GTP-Rac1 and GTP-RhoA which may explain the biphasic regulation of HM-3 and Sunitinib on EAhy926 migration.

## Materials and methods

### Reagents

Sunitinib malate (Sutent, Pfizer) was suspended in solvent 1, which contained carboxymethylcellulose sodium (0.5% w/v), NaCl (1.8% w/v), Tween 80 (0.4%, w/v), benzyl alcohol (0.9 w/v), and deionized water (added to final volume) adjusted to pH 6.0. Peptide HM-3 (Ile-Val-Arg-Arg-Ala-Asp-Arg-Ala-Ala-Val-Pro-Gly-Gly-Gly-Gly-Arg-Gly-Asp) was synthesized by GL Biochem Ltd. (Shanghai, China) and had a purity in excess of 99%. Other reagents included Matrigel (BD Biosciences), Fluorescein Isothiocyanate labeled Phalloidin (Sigma-Aldrich), Rhotekin RBD and PAK-1 PBD agarose conjugates (Millipore). The antibodies used for immunohistochemistry included: anti-CD31 polyclonal antibodies (sc-28188, Santa Cruz Biotech), anti-CD34 polyclonal antibodies (ZA-0550). Docetaxel was from Jiangsu Hengrui Pharmaceutical Co. LTD in China.

RETRACTED

### Cell lines

The human MDA-MB-231-luc^+^ cells were MDA-MB-231 cells co-transfected with a plasmid expressing the firefly luciferase gene (pGL3) and neomycin resistance gene as described previously [5]. These were cultured in minimum essential medium (MEM) with 10% fetal bovine serum (FBS, from Gibco). EAhy926 cells (Shanghai Cell Biology Institutes, Academia Sinica, Shanghai, China) were maintained in RPMI 1640 medium with 10% FBS and antibiotics. B16F10 mouse melanoma cells (Shanghai Cell Biology Institutes, Academia Sinica, Shanghai, China) were maintained in RPMI 1640 medium with 10% FBS (Gibco) and 1% penicillin/streptomycin (Invitrogen, USA). All cells were incubated at 37 °C in 5% CO_2_ in a humidified incubator.

#### Mouse tumor models

BALB/c nude female mice (5–6 weeks, 15-16 g) and C57Bl/6 mice (5–6 weeks, 16-18 g) were purchased from the Shanghai Laboratory Animal Center of the Chinese Academy of Sciences. All animals were housed in a controlled environment (22 ± 2 °C; 12 h light-dark cycle) with water and food provided freely. The experiments involving animals adhered to the ethical standards of China Pharmaceutical University and the care of animals was in accordance with the licensing guidelines of China Pharmaceutical University.

#### Metastasis of human breast cancer MDA-MB-231-luc^+^ cells

After entering logarithmic growth phase, MDA-MB-231-luc^+^ cells were collected and adjusted to a packing of 5 × 10^6^ cells/ml with MEM medium without FBS. 0.2 ml cell suspension was intravenously injected into BALB/c nude mice (two injections of 0.1 ml with a five-minute interval) and the mice were randomly distributed into 5 groups. Mice in group 1 were injected with 0.9% sterilized saline at a dose of 10 ml/kg/day. Mice in group 2 were gavaged with Sunitinib at a dose of 120 mg/kg/d for 7 days from the second day after cancer cell injection. Mice in group 3 were gavaged with Sunitinib at a dose of 60 mg/kg/day during the whole experimental procedure. Mice in group 4 and 5 were intravenously injected with HM-3 at doses of 48 mg/kg/day and 3 mg/kg/day, respectively, during the whole experimental procedure. At day 1, 7 and 21 after cancer cell injection, the bioluminescence of the cancer cells in the lungs or abdomens of the mice were observed with the Caliper IVIS Spectrum system (Massachusetts, USA). Kaplan-Meier survival curves were generated for each group.

RETRACTED

#### Metastasis of mouse B16F10 cells

After entering logarithmic growth phase, B16F10 cells were collected and adjusted to a cell packing of 5 × 10^6^ cells/ml in RPMI 1640 medium without FBS. 0.2 ml cell suspension was intravenously injected into C57BL/6 female mice and the mice were randomly distributed into 5 groups in similar ways as indicated above Mice in group 2 were treated for 7 days, whereas mice in groups 3–5 were treated for 17 days. Mice were sacrificed at day 18. Lung tissues were collected surgically and fixed in 4% formaldehyde. Numbers of metastatic nodules on the lung surfaces of all animals in each group were counted.

#### Histochemistry and immunohistochemistry

Mice from MDA-MB-231-luc + or B16F10 metastasis experiments were sacrificed and lungs were collected, fixed with 4% formaldehyde, embedded in paraffin and sectioned for hematoxylin and eosin (H&E) staining and immunohistochemical staining for CD31 (MDA-MB-231-luc + metastasis experiments) or CD34 (B16F10 metastasis experiments). H&E staining was performed according to standard histological procedures. The presence of cancer cells in lung tissues was observed under a light microscope. Vascular structures in tumors were evaluated after anti-CD31 or anti-CD34 immunostaining with the use of rabbit anti-CD31 or anti-CD34 polyclonal antibodies. Briefly, sections were treated with anti-CD31 or anti-CD34 primary antibody, biotinylated goat anti-rabbit secondary antibody and horseradish peroxidase-labeled streptavidin were added sequentially and visualized by the conversion of the diaminobenzidine (DAB) chromogen. The sections were counterstained with hematoxylin and the tissues were microscopically analyzed. Vascularized areas were identified and viewed at 40 times magnifications. The microvessel density (MVD) of each section was obtained by counting the average number of fifteen fields at 200 times magnification. Three different sections were selected per group.

#### Immunofluorescence

EAhy926 cells were plated onto glass coverslips (NEST Biotechnology) and serum-starved for 12 h after they entered logarithmic growth phase. Control cells were incubated in serum-free culture medium, HM-3 treatment groups were incubated with 4.5 or 17.8 μM HM-3 for 1 h in serum-free cell culture medium, enzyme treatment groups were incubated with PI-PLC (0.5 U/ml) at 30  °C for 30 min before HM-3 treatment. Cells were washed three times with PBS, fixed with 4% paraformaldehyde at 4 °C for 10 min and then blocked with 5% BSA. Cells were then incubated with anti-integrin αvβ3 (SC-7312, Santa Cruz Biotech), or anti-integrin α5β1 (ab75472, Abcam) and anti-Glypican-1 (AF-4519, R&D Systems) antibodies at 4 °C overnight. After washing twice with PBS, cells were incubated with fluorescently labeled secondary antibodies (Alexa Fluor 647 or 488 labeled ab150131 or ab150073, Abcam). Nuclei were counterstained with Hoechst 33342 (H1399, Thermo Fisher Scientific). Images were captured with an OLYMPUS workstation and analyzed with Image J software.

RETRACTED

#### Cell cytoskeleton analysis

Cell cytoskeleton assays were performed as described previously [12]. EAhy926 cells were cultured in gelatin-coated cell culture dishes and serum-starved for 8–12 h before each experiment. Cells were then incubated with Sunitinib (0.015 nM or 2 nM) or HM-3 (4.5 μM or 17.8 μM) at room temperature for 1 h. Subsequently, cells were washed with PBS and fixed with 4% paraformaldehyde at 4 °C for 10 min. Nonspecific protein binding sites were saturated with 5% BSA at room temperature for 30 min. The cells were washed again and then incubated with fluorescein isothiocyanate- (FITC)-labeled Phalloidin for 1 h to visualize the actin cytoskeleton. The cell cultures were finally washed and the fluorescent images were captured using an epifluorescence microscope. The cytoskeleton in MDA-MB-231 cells (cultured in MEM medium) and B16F10 cells (cultured in RPMI 1640 medium) was observed in a similar manner. Cells were treated with Sunitinib (2 or 64 nM) or HM-3 (4.5 or 71.2 μM).

#### Cell proliferation assays

100 μl (3 × 10^4^ cells/ml) EAhy926, B16F10 or MDA-MB-231 cells were added into each well of a 96-well plate. After 12 h, HM-3 or Sunitinib at indicated concentrations and dissolved in serum-free medium were added. Cells in serum-free medium without any drug were used as negative control samples. Docetaxol (12.4 μM) dissolved in serum-free medium was used as a positive control. Endostatin (1 μM) was used as additional positive control, as it has a similar mechanism of action to HM-3. For each concentration 6 replicates were made. After 48 h, 20 μl MTT (5 mg/ml) was added to each well and the plate was incubated at 37 °C for 4 h. Then 100 μl DMSO was added to each well. After gentle shaking, the absorbance of each well was read with a detection wavelength of 570 nm and a reference wavelength of 630 nm. The proliferation inhibitory effect was calculated as (A_negative control_-A_drug_)/A_negative control_× 100%.

RETRACTED

#### EAhy926 migration assay

Transwell experiments were set up as described previously in 24-well plates (Sigma Aldrich) [11]. Matrigel (BD Biosciences) was diluted 1:3 in serum-free Endothelial Cell Medium. 10 μl diluted Matrigel was used to evenly coat the bottom surfaces of the transwells. EAhy926 cells were digested with 0.25% trypsin and resuspended in serum-free Endothelial Cell Medium at a density of 1 × 10^5^ cells/ml. 0.1 ml cell suspension was added to the Matrigel-coated transwells (1 × 10^4^ cells/well). Sunitinib at different concentrations was present in the upper solution. Endostatin (0.4 μM) was used as a positive control. 600 μl Endothelial Cell Medium with 5% FBS and 1% ECGS (endothelial cell growth supplement). The transwells were placed into the 24-well plate and the plate was kept at 37 °C in 5% CO_2_ in an humidified incubator for 24 h. The medium was then aspirated and the migrated cells fixed with ethanol for 30 min. The cells were stained with 0.1% crystal violet for 10 min. The cells that had not migrated were cleared using a cotton swab and microscopic pictures of the migrated cells were taken. Ten photographs were taken for each transwell with three transwells for each experimental condition.

#### Cancer cell invasion assay

Matrigel was diluted 1:2 in serum-free MEM or RPMI 1640 medium. 50 μl diluted Matrigel was used to evenly coat the surface of transwell bottoms. MDA-MB-231 or B16F10 cells were collected and resuspended in serum-free MEM or RPMI 1640 medium at a density of 5 × 10^5^ cells/ml. 0.1 ml cell suspension was added to the Matrigel-coated transwells (5 × 10^4^ cells/well). Sunitinib and HM-3 at different concentrations was present in the upper solution. Endostatin (0.4 μM) was used as a positive control. 600 μl MEM or RPMI 1640 medium with 10% FBS was added to flat-bottoms of the 24-well plates. The transwells were placed into the 24-well plate and the plate was kept at 37 °C in 5% CO_2_ in the humidified incubator for 12 h. Then the transwells were treated and the migrated cells were observed and counted as described above.

#### Flo w cytometry assay

EAhy926 cells were adjusted to a concentration of 1 × 10^6^ cells/ml. Cells were added in a six-well plate with 200 μl cells in each well. For Sunitinib treatment, cells were incubated in the presence of the indicated concentrations of Sunitinib in serum-free medium at 37 °C for 24 h. After washing the cells twice with PBS, cells were collected and incubated with mouse monoclonal anti-VEGFR2 antibody (sc-6251, Santa Cruz) on ice for 1 h. After washing and centrifugation, cells were resuspended and incubated with FITC-labeled goat anti-mouse secondary antibody (ab6785, Abcam) at room temperature for 1 h. After washing twice with PBS, fluorescent signals were collected with MACS Quant Data (Miltenyi Biotec, Germany). Three graphs were created for evaluating the data and creating a gate for the cells. The cells from the control without antibody were analyzed and events gated to remove debris from the analysis. This gate was used for all the samples. For the cell samples, the geometric means of values of events within the gate were calculated. The geometric mean of the control without antibody was subtracted from all of the sample geometric means to remove background noise.

RETRACTED

#### Pull-down assays

Pull-down assays were performed as described previously [15]. EAhy926 cells were treated with Sunitinib (0.015 or 2 nM) or HM-3 (4.45 or 17.8 μM) for 12 h. B16F10 cells were treated with Sunitinib (2 or 64 nM) or HM-3 (4.45 or 71.2 μM) for 12 h. After Sunitinib or HM-3 treatment, cells were lysed in ice-cold lysis buffer (125 mM HEPES, pH 7.5, 750 mM NaCl, 5% NP-40, 50 mM MgCl_2_, 5 mM EDTA, 10% Glycerol, 10 μg/ml leupeptin, 10 μg/ml aprotinin and 1 mM PMSF). The lysates were subsequently incubated with 15 μl agarose beads with Rhotekin RBD (Rho binding domain) or PAK-1 PBD (Rac1 binding domain) at 4 °C for 45 min. Agarose beads (Millipore) were collected by a short centrifugation at 14000 g and resuspended in reducing SDS-PAGE sample buffer. Active forms of extracted Rac1 and RhoA were detected by Western blot with monoclonal antibodies specific for Rac1 (Cell Biolabs) and RhoA (Santa Cruz Biotech).

### Purification of lipid rafts

Buffers. The following buffers were used for the purification of lipid rafts: buffer A (0.25 M sucrose/1 mM EDTA/20 mM Tricine, pH 7.8); buffer B (0.25 M sucrose/6 mM EDTA/120 mM Tricine, pH 7.8); buffer C (50% OptiPrep in buffer B); buffer D (20 mM Tris, pH 7.6/137 mM NaCl/0.5% Tween 20) [28].

Cell culture and drug treatment. 48 flasks of confluent EAhy926 cells were separated into six groups: a control group, a VEGF treatment group (20 ng/ml VEGF for 1 h), two HM-3 treatment groups (4.5 or 17.8 μM HM-3 for 1 h after VEGF induction), or two Sunitinib treatment groups (0.015 or 8 nM Sunitinib for 1 h after VEGF induction). Recombinant human VEGF was from HUMANZYME (HZ-1062).

After drug treatment and washing with PBS, EAhy926 cells in each group were washed twice with 5 ml of buffer A and were collected by scraping in 3 ml of buffer A. After centrifugation (1000 g for 10 min), cell pellets were resuspended in 4 ml buffer A. The cells underwent two rounds of homogenization and centrifugation. Individual supernatants were collected and pooled (total volume around 7 ml). The supernatant was layered on the top of 3 ml of 77% Percoll in buffer A, and centrifuged at 84,000 g for 30 min in a Beckman L-80XP rotor. The visible band of the membrane fraction was collected with a Pasteur pipette, adjusted to 2.0 ml with buffer A and sonicated on ice with two successive bursts (5 s on and 5 s off for 2 min) using a Vibra Cell sonicator (model VC60S, Sonics & Materials, Danbury, CT). Sonicates were mixed with 1.84 ml of buffer C and 0.16 ml of buffer A (final OptiPrep concentration, 23%). A linear 20 to 10% OptiPrep gradient (prepared by diluting buffer C with buffer A) was poured on top of the sample which was then centrifuged at 52,000 g for 90 min in a Beckman L-80XP rotor. The top 2 ml of the gradient (fractions 1–7) were collected, placed in a fresh centrifuge tube, and mixed with 4 ml of buffer C. The sample was overlaid with 2 ml of 5% OptiPrep (prepared by diluting buffer C with buffer A) and centrifuged at 52,000 g for 90 min at 4 °C. A distinct opaque band was present in the 5% OptiPrep overlay about 4–5 mm on the top. This band was collected and designated as lipid raft membranes. Another sample from the bottom 100 μl after centrifugation (84,000 g for 30 min) was sonicated twice and was used as the non-raft sample.

RETRACTED

The raft and non-raft fractions of the samples were analyzed by Western-blot analysis. Primary antibodies included anti-human transferrin R (AF2474, R&D systems), anti-human calveolin (3267, Cell Signaling), anti-integrin αvβ3 (SC-7312, Santa Cruz Biotech), anti-integrin α5β1 (ab75472, Abcam), anti-Glypican-1 (AF-4519, R&D systems), anti-VEGFR2 antibody (sc-6251, Santa Cruz), rabbit monoclonal anti-pVEGFR2 antibody (Y1175) (19A10) (2478S, Cell Signaling). The anti-integrin αvβ3 antibody (SC-7312, Santa Cruz Biotech) was also used for immunoprecipitation.

#### Statistical analysis

Data were analyzed using the statistics software SPSS statistics 17.0 (Softonic, San Francisco, CA, USA) and expressed as mean ± SD. Statistical significance was assessed using the Student *t* test. *p* < 0.05 was considered statistically significant. Higher significance levels (*p* < 0.01) were also indicated.

## Results

### Sunitinib and HM-3 induce biphasic regulation of MDA-MB-231 metastasis and tumor angiogenesis

The MDA-MB-231 metastasis model was established in Balb/c nude mice by intravenous injection of MDA-MB-231-luc^+^ cells and a specific drug treatment protocol (Fig. 1a). The tumor burden was evaluated by bioluminescence detection on day 7 and day 21 after tumor cell injection. 120 mg/kg/d Sunitinib treatment accelerated experimental metastasis (Fig. 1b) and significantly reduced median survival (Fig. 1d, *p* = 0.0216). Representative images are shown in Fig. 1c. Sustained 60 mg/kg/d Sunitinib treatment significantly decreased metastasis (Fig. 1b), though there was not an apparent survival advantage (Fig. 1d, *p* = 0.493 compared with the control group). Similar results were obtained with HM-3. 3 mg/kg/d HM-3 significantly decreased tumor burden (Fig. 1b) and increased median survival (Fig. 1d, *p* = 0.0183). However, 48 mg/kg/d HM-3 significantly increased tumor burden (Fig. 1b) and decreased the median survival rate (Fig. 1d, *p* = 0.0464).

RETRACTED

**Fig. 1:** Effects of Sunitinib and HM-3 on experimental MDA-MB-231 cell metastasis. **a** Treatment protocol of BALB/c nude mice after MDA-MB-231-luc + cells were injected into the tail vein of the mice. **b** Quantification of bioluminescence at day 21 showed accelerated metastasis in groups 2 and 4 compared with the control group, whereas tumor burden was significantly decreased in groups 3 and 5. *p < 0.05, **p < 0.01. **c** Representative images of bioluminescence for each group taken on days 1, 7, and 21 following tumor implantation. **d** Kaplan-Meier survival curves showed significantly decreased median survival of mice in groups 2 and 4 (log-rank test, *p* = 0.0216 and 0.0464) and significant increased median survival of mice in group 5 (*p* = 0.0183). For group 1–5, *n* = 9. **e** Representative examples of micrometastasis in lung by hematoxylin and eosin (H and E) staining (indicated by words in red) and anti-CD31 immunostaining (indicated by words in blue). **f** Statistical analysis of the blood vessel numbers. Results are expressed as mean ± SD (15 regions of three sections per group. *P < 0.05, **P < 0.01 vs. control)

H and E staining and anti-CD31 immunostaining of tumor nodules were performed at day 21. Upon H and E staining (Fig. 1e), larger and more numerous cancer cell clusters were found in the 120 mg/kg/d Sunitinib and 48 mg/kg/d HM-3 treatment groups compared with the controls. By contrast, 60 mg/kg/d Sunitinib and 3 mg/kg/d HM-3 treatment resulted in much fewer cancer cell clusters. As observed after CD31 immunostaining, 120 mg/kg/d Sunitinib and 48 mg/kg/d HM-3 significantly increased blood vessel densities, whereas 60 mg/kg/d Sunitinib and 3 mg/kg/d HM-3 treatment had the opposite effect. These observations were quantified and statistically analyzed on the basis of blood vessel numbers present in tumor tissue slices (Fig. 1f).

### Biphasic regulation of B16F10 metastasis and tumor angiogenesis by Sunitinib and HM-3

The B16F10 metastasis model was established by intravenous injection of tumor cells in C57bl/6 mice. The drug treatment protocol is shown in Fig. 2a. Metastasis of B16F10 cells was evaluated by the number of tumor nodules at the surface of excised lungs. It is apparent from Fig. 2b and c, that 120 mg/kg/d Sunitinib and 48 mg/kg/d HM-3 significantly increased the number of metastatic nodules in groups 2 and 4 whereas 60 mg/kg/d Sunitinib and 3 mg/kg/d HM-3 significantly decreased the nodule numbers compared with the control group. H and E staining and anti-CD34 immunostaining of tumor nodules were performed at day 17. More cancer cell clusters were distributed in lung tissues following 120 mg/kg/d Sunitinib and 48 mg/kg/d HM-3 treatment than in the control group, whereas 60 mg/kg/d Sunitinib and 3 mg/kg/d HM-3 resulted in much fewer cancer cell clusters (Fig. 2d). Anti-CD34 immunostaining showed that 120 mg/kg/d Sunitinib and 48 mg/kg/d HM-3 treatment significantly increased blood vessel density compared with the control group, whereas 60 mg/kg/d Sunitinib and 3 mg/kg/d HM-3 treatment significantly reduced this. Statistical analysis of blood vessel numbers present on tumor nodule slices was executed (Fig. 2e). In both metastasis models, Sunitinib and HM-3 showed a non-linear dose-effect relationship in the regulation of tumor metastasis and tumor angiogenesis.

RETRACTED

**Fig. 2:** Effects of Sunitinib and HM-3 on experimental B16F10 cell metastasis. **a** Treatment protocol of C57BL/6 mice after B16F10 cells were injected via the tail vein. **b** Excised lungs from the experimental B16F10 cell metastasis model were scored visually for surface tumor nodules. **c** Representative images of lungs from different groups at day 17 following tumor implantation. **d** Representative examples of micrometastases in lung by H and E staining (indicated by words in red) and anti-CD34 immunostaining (indicated by words in blue). **e** Statistical analysis of blood vessel numbers. Results are expressed as mean ± SD (15 regions of three sections per group. *P < 0.05, **P < 0.01 vs. control)

As cell proliferation and migration are important processes during angiogenesis and cluster formation of tumor cells, the effects of HM-3 and Sunitinib on these processes were next investigated.

HM-3 also showed a bell-shaped dose-effect curve in inhibition of primary tumor growth in nude mice (Additional file 1: Figure S1-S3, Additional file 1: Table S1-S4, S6). The other anti-angiogenic drugs with a special dose-effect curve was shown in Additional file 1: Table S5.

### Regulation of cell proliferation by HM-3 and Sunitinib

MTT assays were performed to evaluate the effect of HM-3 and Sunitinib on EAhy926, B16F10 and MDA-MB-231 proliferation. In all cases, the positive control (Docetaxol, 12.4 μM) showed more than 90% inhibition of cell proliferation. Endostatin (ES, 1 μM), which has a similar mode of action to HM-3, induced a 40% inhibition of EAhy926s cell proliferation but did not inhibit the proliferation of B16F10 and MDA-MB-231 cells (Fig. 3a-f). HM-3 dose-dependently inhibited EAhy926 proliferation (Fig. 3a). However, the inhibition was relatively inefficient, and even at 144 μM the inhibition rate was only 34%. HM-3 did not inhibit the proliferation of B16F10 and MDA-MB-231 cells (Fig. 3b and c). Sunitinib dose-dependently inhibited the proliferation of EAhy926, B16F10 and MDA-MB-231 at the micromolar level with a similar inhibition profile (Fig. 3d-f). The different inhibition profiles of Docetaxol, ES, HM-3 and Sunitinib were well correlated with their mechanisms of action.

RETRACTED

**Fig. 3:** **a**-**c** Inhibition of HM-3 in the proliferation of EAhy926 (**a**), B16F10 (**b**) and MDA-MB-231 (**c**) cells. **d**-**f** Inhibition of Sunitinib in the proliferation of EAhy926 (**d**), B16F10 (**e**) and MDA-MB-231 (**f**) cells.

### EAhy926 migration and B16F10 and MDA-MB-231 invasion show non-linear concentration effect relationship

In previous studies, HM-3 displayed a bell-shaped concentration-effect curve in regulation of EAhy926 migration [11]. HM-3 was found to inhibit EAhy926 migration between 0.14 to 4.5 μM in a concentration-dependent way, but further increases in HM-3 concentration resulted in reduced inhibition or even promotion of EAhy926 cell migration [13]. We therefore investigated the regulation of EAhy926 migration by Sunitinib (migrating cell numbers shown in Fig. 4b and migration inhibition rates shown in Fig. 4c). Typical photographs of the bottoms of the transwells under each experimental condition were shown in Fig. 4a. As observed for HM-3, Sunitinib at a low concentratin (e.g. 0.015 nM) significantly inhibited EAhy926 migration whereas at higher concentrations (e.g. 8 or 32 nM), Sunitinib promoted EAhy926 migration. The effects of Sunitinib and HM-3 on MDA-MB-231 and B16F10 invasion were also evaluated. Bell-shaped concentration-effect curves were found for both cell lines for both reagents (Fig. 4d-g). 0.015 and 2 nM Sunitinib significantly inhibited B16F10 (Fig. 4d) and MDA-MB-231 (Fig. 4f) invasion whereas 64 nM Sunitinib significantly promoted the invasion of MDA-MB-231 and B16F10 cells. Similarly, 4.5 μM HM-3 inhibited invasion of B16F10 and MDA-MB-231 cells (Fig. 4e and g) whereas 71 μM HM-3 resulted in significantly enhanced invasion in both cell lines.

**Fig. 4:** Regulation of EAhy926 cell migration and B16F10 and MDA-MB-231 cell invasion by HM-3 and Sunitinib. EAhy926 cell migration and B16F10 and MDA-MB-231 cell invasion were assayed using the transwell method. 0.1 ml EAhy926 cell suspension (1 × 10^5^ cells/ml), B16F10 cell suspension (5 × 10^5^ cells/ml) or MDA-MB-231 (5 × 10^5^ cells/ml) cell suspension were added to Matrigel-coated transwells. HM-3 or Sunitinib were present in the upper solution at different concentrations. Endostatin (ES, 0.4 μM) was used as a positive control reagent. The cell migration tests were performed at 37 °C for 24 h. **a** Typical microphotographs of the migrated EAhy926 cells in the presence of Sunitinib at indicated concentrations. Migrated cells are colored purple, while cells without migration are transparent. Numbers of migrated cells (**b)** and percent inhibition of migration (**c)** are shown. Percent inhibition by Sunitinib (**d)** and HM-3 (**e)** in B16F10 cell invasion. Percent inhibition of Sunitinib (**f**) and HM-3 (**g**) in MDA-MB-231 cell invasion. In each case, HM-3 or Sunitinib inhibited cell migration or invasion at low doses and promoted cell migration or invasion at high doses (*P < 0.05, **P < 0.01)

From the data in both Figs. 3 and 4 we concluded that HM-3 and Sunitinib did not efficiently inhibit EAhy926 and tumor cell proliferation, whereas they efficiently regulated EAhy926 cell migration and tumor cell invasion with non-linear concentration-effect relationships. The molecular mechanisms for regulation of cell migration and invasion were therefore further investigated.

RETRACTED

Pharmacokinetics study of HM-3 in rats was performed. It was found that serum HM-3 levels in rats were on a nanomolar level after an intravenous injection of 2.1 mg/kg HM-3 and this level decreased quickly (Additional file 1: Figure S4, Additional file 1: Table S7-S8). Levels of HM-3 in lung, liver, heart and muscle within 60 min after HM-3 injection remained around 10 ng/ml (5.6 nM) and HM-3 levels in the other organs were lower than 1 ng/ml (Additional file 1: Figure S5, Additional file 1: Table S9). It is possible that though the whole HM-3 molecule in mouse blood is not stable, its fragments that contain the central part of ES-2 and RGD sequence can still act on their targets and biologically active as has been found in another peptide P2 (Additional file 1: Figures S6-S7).

Binding of FITC labeled HM-3 to integrin expressing cells was tested with a flow cytometry method and the rate of cells with positive fluorescence signal was measured (Additional file 1: Figure S8 and S9, and Additional file 1: Table S10). The concentration of FITC-HM-3 in this experiment is 1 μg/ml or 0.46 μM, which is lower than the 4.5 μM for HM-3 to inhibit endothelial cell migration and tumor cell invasion (Fig. 4).

### Regulation of the levels of active forms of RhoA and Rac1 by Sunitinib and HM-3

RhoGTPases are central regulators of cell migration. Rhotekin RBD (Rho binding domain) or PAK-1 RBD (Rac1 binding domain), respectively, were used to extract active forms of Rac1 or RhoA from EAhy926 cell lysates after the cells had been treated with different concentrations of Sunitinib or HM-3. The levels of the active forms of RhoA and Rac1 within EAhy926 cells (Fig. 5a and b) and B16F10 cells (Fig. 5c and d) after cell treatment under different conditions were investigated by extraction from cell lysates with agarose beads and analysis by Western-blot. Again, a non-linear concentration-effect relationships were found. Sunitinib at 0.015 nM and 4.5 μM HM-3 both decreased the amounts of GTP-Rac1 and GTP-RhoA within EAhy926 cells whereas 8 nM Sunitinib and 18 μM HM-3 treatments substantially increased these levels (Fig. 5a and b). As GTP-Rac1 and GTP-RhoA activities are essential for cell movement [14], the changes of GTP-Rac1 and GTP-RhoA observed in EAhy926 cells were in line with the expectations. Similarly, by the data in Fig. 5c and d it was illustrated that 2 nM Sunitinib and 4.5 μM HM-3 both decreased the levels of GTP-Rac1 and GTP-RhoA in B16F10 cells whereas 64 nM Sunitinib and 71 μM HM-3 increased these levels.

RETRACTED

**Fig. 5:** Effects of Sunitinib and HM-3 on the levels of the active form of RhoGTPases and cytoskeleton within the target cells. **a**-**d** To test the levels of active form RhoGTPases in EAhy926 cells, Rhotekin RBD (Rho binding domain) or PAK-1 PBD (Rac1 binding domain) were used to extract active form Rac1 (**a**) or RhoA (**b**) from EAhy926 cell lysates after the cells were treated with different concentrations of Sunitinib or HM-3 as indicated. Immunoblotting was performed with specific Rac1 or RhoA antibodies. Cells that had not been treated were used as a positive control. The levels of GTP-Rac1 (**c**) and GTP-RhoA (**d**) in B16F10 cells were assayed in an analogous way. Quantification of GTP-Rac1 or GTP-RhoA signal ratios is indicated. **e** Effect of Sunitinib and HM-3 on the EAhy926 cytoskeleton. The images for cytoskeleton of EAhy926, B16F10 or MDA-MB-231 cells were indicated with black, red or blue words respectively. For EAhy926 images, cells were treated with 0.015 or 8 nM Sunitinib, 4.5 or 17.8 μM HM-3 at room temperature for 1 h. After fixation, nonspecific binding sites were saturated with 5% BSA. Fluorescein isothiocyanate labeled phalloidin was used to visualize actin stress fibers. For B16F10 and MDA-MB-231 images, cells were treated with 2 nM or 64 nM Sunitinib, 4.5 μM or 71 μM HM-3 at room temperature for 1 h. Cells that had not been treated were used as a control

Cell morphology was related to the RhoGTPase activities. Intact EAhy926 cells in the control group displayed abundant actin stress fibers across the cells (Fig. 5e). In EAhy926 cells treated with 0.015 nM Sunitinib or 4.5 μM HM-3, the network of actin stress fibers was less extensive than in the control cells and was restricted to the cell peripheries, which is consistent with the observed lower RhoA activities (Fig. 5b), and the concept that cell migration was inhibited by the absence of stress fiber constriction. In the EAhy926 cells that were treated with 8 nM Sunitinib or 17.8 μM HM-3, more stress fibers were displayed with branching structures extending out. The morphological appearance of MDA-MB-231 and B16F10 cells after Sunitinib and HM-3 treatment is shown in Fig. 5c. The intact cells in the control group displayed abundant actin stress fibers across the cells. In cells treated with 2 nM Sunitinib or 4.5 μM HM-3 the amounts of actin stress fibers were significantly reduced and the cells had smooth borders. In cells treated with 64 nM Sunitinib or 71.2 μM HM-3, more actin stress fibers were present with branching structures extending out.

RETRACTED

It has been reported that endostatin can recruit its target, integrin α5β1, to lipid rafts by simultaneous interaction with glypican-1 that only exists in this region [15]. ES-2 covers one of the two active domains of endostatin that binds to heparin and inhibits FGF-2- and VEGF-A-induced chemotaxis of endothelial cells [29]. It was of interest to investigate if the regulation of HM-3 in EAhy926 migration is glypican-1- and lipid raft-dependent and whether Sunitinib shared a similar or different mechanism.

### Regulation of EAhy926 migration by HM-3 depends on glypican-1

To investigate if the regulatory effects of an effective concentration (e.g. 4.5 μM) or a higher one (e.g. 17.8 μM) of HM-3 were glypican-1- dependent, EAhy926 cells were treated with 5 U/ml Heparinase I (Hep I) or 0.5 U/ml phosphatidylinositol-.

phospholipase C (PI-PLC) before the migration assays. Hep I cleaves the proteoglycan side-chains of glypican-1 while PI-PLC can remove glypican-1 by cleavage of phosphatidylinositol. Migration as evaluated by cell numbers and the corresponding inhibition rates were obtained (Fig. 6a and b). With the use of control samples we confirmed that neither Hep I nor PI-PLC treatment had any obvious effect on EAhy926 migration (Fig. 6a). Without enzyme pre-treatment, 4.5 μM HM-3 significantly decreased migrating cell numbers compared with the corresponding control samples. By contrast, both 5 U/ml Hep I or 0.5 U/ml PI-PLC pretreatment increased migrating cell numbers compared with the samples treated with peptide. Migration inhibition rates were calculated. The inhibitory effect of 4.5 μM HM-3 on EAhy926 cell migration was 50% and after enzyme pretreatment, this inhibitory effect was substantially decreased (Fig. 6b). By contrast, 17.8 μM HM-3 promoted EAhy926 migration by 20% and after Hep I or PI-PLC treatments, HM-3 generated strong inhibition of EAhy926 cell migration (Fig. 6b). with these results we indicated that the regulatory effect of HM-3 in EAhy926 migration is heparan sulfate proteoglycan-dependent. As only glypicans anchor to the cell surface via phosphatidylinositol (whereas syndecans do not), the fact that PI-PLC pretreatment decreased the inhibitory effect of AP25 on EAhy926 migration was in line with the idea that the heparin sulfate proteoglycan (as a co-receptor for AP25) belongs to the glypcian family.

RETRACTED

**Fig. 6:** HM-3 regulated EAhy926 migration in a glypican-1 dependent manner. **a** and **b** EAhy926 cells were left untreated or treated with 5 U/ml Hep I or 0.5 U/ml PI-PLC and cell migration assays were performed in the presence of 4.5 or 17.8 μM HM-3. 0.4 μM Endostatin (ES) was used as a positive control. Untreated or enzyme treated cells without peptide treatment were used as controls. The migrating cell numbers for each condition are shown in panel **a** and the migration inhibition rate in panel **b**. **c**-**f** Integrin αvβ3 and α5β1 co-localize with glypican-1. Integrin αvβ3 (**c**) and α5β1 (**e**) on cell surface are shown in green (Alexa Fluor 488) and glypican-1 in red (Alexa Fluor 647). Nuclei were counterstained with Hoechst 33342. Images were captured with an OLYMPUS workstation and analyzed with Image J software. Histograms for co-localization of integrin αvβ3 (**d**) or α5β1 (**f**) with glypican-1 as calculated by the intensities of the merged signals (*P < 0.05, **P < 0.01)

### Integrin α5β1 and αvβ3 co-localize with glypican-1

Immunofluorescence detection of integrin α5β1 and αvβ3 at the cell surface was used to investigate whether these integrins colocalize with glypican-1, the major glypican expressed on endothelial cells [30]. From Fig. 6c and e it was deduced that an obvious correspondence of the signals for the integrins and glypican-1 existed in control cells. After 4.5 or 17.8 μM HM-3 treatment, the intensities of merged signals increased dose-dependently, but after PI-PLC treatment the glypican-1 signal virtually disappeared. Treatment with 4.5 or 17.8 μM HM-3 did not change the signals for integrin α5β1 and αvβ3 and the signals for co-localization of the integrins and glypican-1 were almost undetectable. Percentages of integrin accumulation in lipid rafts were calculated (Fig. 6d) for integrin αvβ3 and for integrin α5β1 (Fig. 6f). Our data confirmed that integrin α5β1 and αvβ3 co-localized with glypican-1. As glypican-1 only exists in the lipid raft region [15], we further investigated whether integrin α5β1 and αvβ3 are recruited into lipid rafts after HM-3 or Sunitinib treatments.

RETRACTED

### Distribution of integrin α5β1, αvβ3 and VEGFR2 in raft and non-raft regions after HM-3 and Sunitinib treatment

Raft and non-raft regions were separated and collected with the use of a detergent- free centrifugation method [28]. The distribution of integrin α5β1, αvβ3 and VEGFR2 in the raft and non-raft regions was analysed by comparison of their levels on Western-blot. As described in Material and Methods, following three centrifugation steps, the upper layer (around 1.0 ml) was collected as the raft region. The lower layers after the second and third centrifugation were combined as the membrane fraction outside of the raft region (non-raft region) (Fig. 7a). Human transferrin R and caveolin-1, respectively, were used as a non-raft marker and a raft marker. As shown in Fig. 7b, there was no apparent cross contamination of the membrane fractions of the raft and non-raft regions. Additionally, glypican-1 was only found in the lipid raft region, which is in agreement with previous reports [15]. Integrin α5β1 and αvβ3 existed in both the raft and non-raft regions (Fig. 7c). Distribution of integrin α5β1 and αvβ3 after HM-3 and Sunitinib treatments are shown in Fig. 7d and e. After HM-3 treatment, the levels of both integrin α5β1 and αvβ3 inside the lipid raft region significantly increased. More integrin α5β1 and αvβ3 accumulated inside the lipid raft region following treatment with 17.8 μM HM-3 than with 4.5 μM (Fig. 7d and e, left panel). Additionally, treatment with Sunitinib also recruited integrin α5β1 and αvβ3 to the lipid raft region (Fig. 7d and e, right panel).

**Fig. 7:** Distribution of integrin α5β1, αvβ3 and VEGFR2 on EAhy926 cell surface after HM-3 and Sunitinib treatment. **a** Treatment strategy. Samples 1–6 are membrane fractions outside of the lipid raft region and samples 7–12 are membrane fractions inside the lipid raft region of the corresponding cells. **b** Detection of human transferrin R (non-raft marker) and caveolin-1 (raft marker) with Western-blot analysis. Glypican-1 was also analysed. **c** Western-blot analysis showing redistribution of integrin α5β1 and αvβ3 after HM-3 and Sunitinib treatment. Intensities of the protein bands were analyzed with Image J and shown as histograms in panel **d** for integrin α5β1 and panel **e** for integrin αvβ3. Statistical analysis was performed with VEGF induced samples (sample 2 and 8) for comparison of non-raft and raft fractions. **f** Western-blot analysis showing redistribution of VEGFR2 and p-VEGFR2 after HM-3 and Sunitinib treatment. Intensities of the protein bands were shown as histograms in panel **g** for VEGFR2 and panel **h** for p-VEGFR2. Statistical analysis was performed comparing sample 2 or 8. **i** Immunoprecipitation was performed with anti-integrin αvβ3 antibodies and VEGFR2 or p-VEGFR2 was detected with Western-blot analysis to show distribution of integrin αvβ3-VEGFR2 complexes and the corresponding p-VEGFR2. Intensities of the protein bands were analyzed with Image J and shown as histograms in panel **j** for VEGFR2 and panel **k** for p-VEGFR2. Statistical analysis was performed comparing sample 2 for the non-raft region and sample 8 for the raft region. Data are represented as mean ± SD (*p<0.05, **p<0.01)

The distribution of VEGFR2 and p-VEGFR2 after HM-3 and Sunitinib treatments was also investigated (Fig. 7f) and band densities were analyzed (Fig. 7g and h). After HM-3 treatment, the amounts of VEGFR2 and p-VEGFR2 inside the lipid raft region both significantly increased, with higher levels found with 17.8 μM compared with 4.5 μM treatment (Fig. 7g and h, left panel). Sunitinib also recruited VEGFR2 and p-VEGFR2 to the lipid raft region with a significant difference (Fig. 7g and h, right panel). As integrin αvβ3 and VEGFR2 were both recruited to the lipid raft region and their interactions and cross activations are reported previously [25], immunoprecipitation reactions were performed to detect the presence of integrin-VEGFR2 complexes and their distribution after HM-3 and Sunitinib treatments. VEGFR2 protein was not detected after immunoprecipitation with anti-integrin α5β1 antibodies. However, clear VEGFR2 and the corresponding p-VEGFR2 proteins were found after immunoprecipitation with anti-integrin αvβ3 antibodies (Fig. 7i). In control cells without VEGF induction, only basal levels of integrin αvβ3-VEGFR2 complex were observed. After VEGF induction, levels of this complex increased significantly (Fig. 7j and k). After 4.5 or 17.8 μM HM-3 treatment, the amounts of integrin αvβ3-VEGFR2 complex and p-VEGFR signals in the non-raft region significantly decreased and those in the raft region significantly increased (Fig. 7j and k). Under Sunitinib treatment, the amounts of integrin αvβ3-VEGFR2 complex and p-VEGFR signals in raft regions also significantly increased, although the increases were less than those observed with HM-3.

RETRACTED

Raft region isolation and collection was also performed after glypican-1 cleavage (Fig. 8). Sample treatment strategies are shown in Fig. 8a. Lipid rafts were successfully isolated and no cross contamination of raft and non-raft regions was observed (Fig. 8b). After PI-PLC treatment, the signal for glypican-1 in the lipid raft region disappeared (Fig. 8b). After VEGF induction, the amounts of integrin α5β1 and αvβ3 increased in samples 2 and 8 (compared with samples 1 and 7) whereas these amounts decreased in both raft and non-raft regions after treatment with 4.5 or 17.8 μM HM-3 (Fig. 8c). For both integrins, levels in the non-raft region showed a significant decrease after HM-3 and Sunitinib treatments. The levels of integrin α5β1 in the lipid raft region decreased after treatment with 17.8 μM HM-3 or 8 nM Sunitinib, whereas there was no significant change in the amounts of integrin αvβ3 (Fig. 8d and e). Distribution of VEGFR2 and p-VEGFR2 under HM-3 and Sunitinib treatment after glypican-1 cleavage were also investigated (Fig. 8f) and band densities, as a measure of protein levels, were analyzed (Fig. 8g and h). In the lipid raft region, the signals for VEGFR2 and p-VEGFR2 were substantially decreased by 17.8 μM HM-3 or 8 nM Sunitinib treatments. Both HM-3 and Sunitinib treatments decreased the amounts of VEGFR2 and p-VEGFR2 outside of the lipid raft region. In general, after glypican-1 cleavage, the signals for integrins, VEGFR2 and p-VEGFR2 inside the lipid raft region were substantially decreased and lower than those outside of the lipid raft region (Fig. 8c-h). Levels of integrin αvβ3-VEGFR2 complex under different conditions were detected by immunoprecipitation and Western-blot analysis (Fig. 8i, j and k). The amounts of integrin αvβ3-VEGFR2 complex and the corresponding p-VEGFR2 in the lipid raft region were much lower than outside, which was in contrast with the results in Fig. 7i, j and k. As this complex formation and its cross activation are important for RhoGTPase activation and cell migration [25], these data are in line with the cell migration assay in Fig. 6b and explain why 17.8 μM HM-3 strongly inhibited EAhy926 migration after glypican-1 cleavage.

**Fig. 8:** Distribution of integrin α5β1, αvβ3 and VEGFR2 on EAhy926 cells by HM-3 and Sunitinib treatment after cleavage of glypican-1. **a** Treatment strategy. Samples 1–6 are membrane fractions outside of the lipid raft region and samples 7–12 are membrane fractions inside the lipid raft region of the corresponding cells. **b** Detection of human transferrin R (non-raft marker) and caveolin-1 (raft marker) with Western-blot analysis. The distribution of glypican-1 was also analyzed. **c** Western-blot analysis to show redistribution of integrin α5β1 and αvβ3 by HM-3 and Sunitinib treatment after glypican-1 cleavage. Intensities of the protein bands were analyzed with Image J and shown as histograms in panel **d** for integrin α5β1 and panel **e** for integrin αvβ3. Statistical analysis was performed to samples 2 and 8. **f** Western-blot analysis to show distribution of VEGFR2 and p-VEGFR2 by HM-3 and Sunitinib treatment after glypican-1 cleavage. Intensities of the protein bands were shown as histograms in panel **g** for VEGFR2 and panel **h** for p-VEGFR2. Statistical analysis was performed to compare samples 2 and 8. **i** Immunoprecipitation was performed with anti-integrin αvβ3 antibodies and VEGFR2 or p-VEGFR2 was detected with Western-blot analysis to show distribution of integrin αvβ3-VEGFR2 complexes and the corresponding p-VEGFR2 on glypican-1-cleaved cells. Intensities of the protein bands were analyzed with Image J and shown as histograms in panel **j** for VEGFR2 and panel **k** for p-VEGFR2. Statistical analysis was performed comparing sample 2 for the non-raft region and sample 8 for the raft region. Data are represented as mean ± SD (*p<0.05, **p<0.01)

In general, the signals for integrins, VEGFR2 or p-VEGFR2 inside the lipid raft region in intact cells were higher than those outside of the lipid raft region (Fig. 7). After glypican-1 cleavage, the signals for these molecules were substantially decreased and lower than those outside of the lipid raft region (Fig. 8).

RETRACTED

### Expression of VEGFR2 on EAhy926 surface after Sunitinib treatments

Norton et al. reported that treatment with Sunitinib at micromolar levels for 1.5 h specifically increased VEGFR2 on the MEC (microvascular endothelial cells) cell surface [31]. We therefore used flow cytometric analysis (Fig. 9) to determine the level of VEGFR2 on EAhy926 cells under the same treatment conditions used for the EAhy926 migration assays (Fig. 4c). Untreated cells were used to control for background fluorescence (Panel a). Histograms for cells incubated without or with different concentrations of Sunitinib are shown in panels b-f. It can be seen (panel g) that Sunitinib at 0.015 or 0.03 nM significantly decreased levels of VEGFR2 whereas 5 or 32 nM Sunitinib caused a significant increase. As VEGFR2 is the main receptor mediating VEGF-induced cell migration, this result was in line with the Sunitinib mediated EAhy926 cell migration assays (Fig. 4c).

**Fig. 9:** Effect of Sunitinib on the levels of VEGFR2 on EAhy926 surface**.** EAhy926 cells were incubated with Sunitinib at indicated concentrations at 37 °C for 24 h. Cells were incubated with anti-VEGFR2 antibody followed by FITC labeled secondary antibody. **a** VEGFR2 numbers for a no-antibody control was generated and the geometric mean calculated. This was used to control for background fluorescence. Histograms showing the number of VEGFR2 for the untreated (0 μM Sunitinib) (**b**) and treated (**c-f**) EAhy926 cells were generated, and the geometric mean calculated. **g** Comparison of the geometric mean of Sunitinib treated cells with the control (0 μM Sunitinib) sample (*p<0.05, **p<0.01)

RETRACTED

## Discussion

Sunitinib and HM-3 have different molecular targets and belong to different classes of anti-angiogenic agents. They both inhibited tumor metastasis and tumor angiogenesis at specific doses but promoted these processes at higher doses in two independent animal models: metastasis of B16F10 cells in syngeneic mice and metastasis of human MDA-MB-231 cells in nude mice (Figs. 1 and 2). These effects were independent of the immune regulatory system and different tumor microenvironments. Both Sunitinib and HM-3 have also been reported to inhibit angiogenesis in a model of collagen-induced arthritis [32, 33]. Their anti-angiogenic effects therefore appear to be broadly applicable.

HM-3 showed a limited inhibition of EAhy926 cell proliferation and it did not inhibit tumor cell proliferation (Fig. 3). HM-3 inhibited cell migration at 4.5 μM,whereas it promoted cell migration at 18 μM (Fig. 4). This is in line with a previous report that endostatin, a molecule that targets integrin αvβ3 and α5β1, exerted its anti-angiogenic activity by inhibition of endothelial cell migration [15]. Sunitinib at concentrations more than 3.1 μM inhibited cell proliferation in a dose dependent way (Fig. 3) whereas it regulated cell migration at nanomolar levels. Sunitinib inhibited EAhy926 cell migration and tumor cell invasion at 0.015 and 2 nM and it significantly promoted these processes at 8 or 64 nM (Fig. 4). As HM-3 and Sunitinib regulated cell migration at low concentrations with a non-linear dose-effect relationship that was similar to their regulation of tumor metastasis and tumor angiogenesis, the molecular mechanism for the regulation of EAhy926 cell migration was further investigated.

Integrin distribution in either the raft or non-raft region appeared to explain how HM-3 and Sunitinib regulate endothelial cell migration. Integrin interactions with their ligands regulate the activities of intracellular RhoGTPases, which are central regulators of cell migration [34]. They form a complex with the Src family of tyosine kinases (SFKs) located downstream of integrins [35] and regulate the activities of GEFs and GAPs that act on RhoGTPases. For instance, integrin engagement can induce the formation of the FAK-Src complex [21], which activates the GEF for Rac1 [36, 37] and Cdc42 [37], and activates GAP [38] and GEF [39, 40] for RhoA. On the other hand, growth factor receptors can be recruited to sites of integrin ligation [41] promoting phosphorylation and controling RhoGTPases through direct interactions with GEFs or GAPs [42]. HM-3 and Sunitinib treatments both increased the levels of integrin α5β1 and αvβ3 in the lipid raft region (Figs. 7 and 8). Wickström showed that endostatin recruits in a glypican-1-dependent way integrin α5β1 into the lipid raft region resulting in decreased RhoA activity by Src dependent activation of p190RhoGAP, thereby inhibiting endothelial cell migration [15]. We have further confirmed that not only integrin α5β1 but also αvβ3 can be recruited into the lipid raft region. While HM-3 recruits these integrins into the lipid raft region by interactions with glypican-1, the mechanism by which Sunitinib achieved these recruitments remain unclear. Additionally, the distribution of VEGFR2 and p-VEGFR2 inside or outside of the lipid raft region under HM-3 and Sunitinib treatments was similar to that of integrin α5β1 and αvβ3 (Fig. 7F to H). With immunoprecipitation experiments we found that under HM-3 and Sunitinib treatments, the levels of integrin αvβ3-VEGFR2 complex in the lipid raft region substantially increased, especially under HM-3 treatment. As integrin αvβ3 and VEGFR2 interactions promote VEGFR2 activation (Fig. 7k) and RhoGTPase activitiy (Fig. 5a-d), this may explain how high dose HM-3 and Sunitinib can promote EAhy926 cell migration. We hypothesized that 4.5 μM HM-3 inhibited EAhy926 migration mainly by integrin α5β1 engagement of the ES-2 region whereas at 17.8 μM HM-3 promoted EAhy926 cell migration mainly by RGD interactions with integrin αvβ3 and the formation of αvβ3-VEGFR2 complex in the lipid raft region (Fig. 10). After glypican-1 cleavage, the signals for integrins and αvβ3-VEGFR2 complex in the lipid raft region were all substantially decreased and lower than the signals outside of lipid raft region (Fig. 8). Salanueva et al. have reported that with cells in suspension, lipid raft domains were rapidly endocytosed by a mechanism involving translocation of pYCav-1 from the intracellular region of integrins to the lipid raft domain [43]. It is possible that, following glypican-1 cleavage, integrin α5β1 and αvβ3 outside of lipid raft region can interact with freely moving ligand (e.g. HM-3) and that 17.8 μM HM-3 treatment may induce endocytosis of the lipid raft region so that the levels of integrins and αvβ3-VEGFR2 complex inside the lipid raft region are now lower than those outside. This can explain the strong inhibitory effect of 17.8 μM HM-3 after glypican-1 cleavage (Fig. 6b).

RETRACTED

**Fig. 10:** Mechanisms of Sunitinib and HM-3 actions

Sunitinib also regulated the amounts of integrin α5β1, αvβ3 and VEGFR2 inside or outside of the lipid raft regions. Norton et al. reported that 1 μM Sunitinib treatment of MEC for 1.5 h specifically increased levels of VEGFR2 on the MEC cell surface whereas the number of VEGFR1 remained constant [31]. To better understand the results of our cell migration assays, we therefore used nanomolar concentrations of Sunitinib and incubated EAhy926 cells for 24 h instead of 1.5 h. We found that Sunitinib biphasically regulated the number of VEGFR2 at the EAhy926 cell surface (Fig. 9). After enzyme cleavage of glypican-1, the signals for integrin α5β1, αvβ3 and VEGFR2 in lipid raft region all decreased and were lower than those outside of lipid raft region, indicating that HM-3 and Sunitinib regulated the distribution of these molecules in a glypican-1 related manner.

## Conclusions

Currently, Sunitinib is in clinical use and HM-3 has entered clinical trials. However, dose-effect relationships need to be carefully monitored. The use of higher than the effective dose may cause lower efficacy or even the reversed effect. To our knowledge this is the first time that anti-angiogenic reagents with different working mechanisms have been compared and their general regulatory effect on tumor metastasis was investigated and confirmed. Our work suggested that effective treatment may only be achieved within a strict dose window. This study provides useful guidelines for future clinical applications of anti-angiogenic drugs.

## Additional file

Additional file 1: **Figure S1.** Effect of effective dose or high dose HM-3 on the growth of subcutaneous A549 cells in nude mice. **Figure S2.** Effect of effective dose or high dose HM-3 on the growth of subcutaneous A549 cells in nude mice. **Figure S3.** Effect of effective dose or high dose HM-3 and Sunitinib on the growth of subcutaneous HT29 cells in nude mice. **Figure S4.** A serum HM-3 concentration versus time curve after a single intravenous injection of 2.1 mg/kg HM-3 in rats. **Figure S5.** Tissue distribution of HM-3 after a single intravenous injection of 2.1 mg/kg HM-3 in rats. **Figure S6.** Sequence and domains of peptide HM-3 and P2. **Figure S7.** Levels of peptide P2 in mouse serum after a single intravenous injection of 30 mg/kg P2 and residue inhibitory activity of P2 in MMP-2 activity. **Figure S8.** Western blot detection of the expression of integrin αv, α5, β3, β1 subunit and VEGFR2 on HUVEC, A549, MCF-7, Hela, BEL-7402, MGC-803, HT-29, MDA-MB-435 and U87 cells. **Figure S9.** Flow cytometry analysis to detect the binding of FITC-HM-3 on HUVEC. **Table S1.** Drug treatment strategy for A549 transplant model in nude mice in which drug treatment started when tumor grew to 70 mm^3^. **Table S2.** Drug treatment strategy for A549 transplant model in nude mice in which drug treatment started when tumor grew to 130 mm^3^. **Table S3.** Drug treatment strategy for A549 transplant model in nude mice in which drug treatment started when tumor grew to 300 mm^3^. **Table S4.** Drug treatment strategy for HT29 transplant model in nude mice in which drug treatment started when tumor grew to 75 mm^3^. **Table S5.** Anti-angiogenic drugs with a special dose-effect relationship. **Table S6.** Growth inhibition rates based on tumor weight on day 21 of the four animal experiments as presented in Table S1-S4 and Figure S1-S3. **Table S7.** Serum concentrations of HM-3 in rats after a single intravenous injection of 2.1 mg/kg HM-3. **Table S8.** Pharmacokinetic parameters in rats after a single intravenous injection of 2.1 mg/kg HM-3. **Table S9.** Tissue distribution of HM-3 in rats after a single intravenous injection of 2.1 mg/kg HM-3. **Table S10.** Binding rates of FITC-HM-3 on various types of cells. (DOCX 487 kb)

RETRACTED

## Data Availability

All data generated or analysed during this study are included in this published article [and its supplementary information files].

## Abbreviations

FAK: Focal adhesion kinase
GAP: GTPase-activating proteins
GEF: Guanine nucleotide exchange factor
GPI: Glycosylphosphatidylinositol
Hep I: Heparinase I
PI-PLC: Phosphatidylinosital-phospholipase C
Src: Src family kinase

## References

[1] Folkman J (1971). Tumor angiogenesis: therapeutic implications. N Engl J Med.

[2] Demetri GD, van Oosterom AT, Garrett CR, Blackstein ME, Shah MH, Verweij J (2006). Efficacy and safety of sunitinib in patients with advanced gastrointestinal stromal tumor after failure of imatinib: a randomised controlled trial. Lancet.

[3] Motzer RJ, Michaelson MD, Redman BG, Hudes GR, Wilding G, Figlin RA (2006). SU11248, a multitargeted inhibitor of vascular endothelial growth factor receptor and platelet-derived growth factor receptor, in patients with metastatic renal cell carcinoma. J Clin Oncol.

[4] Pàez-Ribes M, Allen E, Hudock J, Takeda T, Okuyama H, Viñals F (2009). Antiangiogenic therapy elicits malignant progression of tumors to increased local invasion and distant metastasis. Cancer Cell.

[5] Ebos JM, Lee CR, Cruz-Munoz W, Bjarnason GA, Christensen JG, Kerbel RS (2009). Accelerated metastasis after short-term treatment with a potent inhibitor of tumor angiogenesis. Cancer Cell.

[6] Brahimi-Horn MC, Chiche J, Pouysségur J (2007). Hypoxia and cancer. J Mol Med.

[7] Grunewald M, Avraham I, Dor Y, Bachar-Lustig E, Itin A, Jung S (2006). VEGF-induced adult neovascularization: recruitment, retention, and role of accessory cells. Cell..

RETRACTED

[8] Ebos JM, Lee CR, Christensen JG, Mutsaers AJ, Kerbel RS (2007). Multiple circulating proangiogenic factors induced by sunitinib malate are tumor-independent and correlate with antitumor efficacy. Proc Natl Acad Sci U S A.

[9] Mendel DB, Laird AD, Xin X, Louie SG, Christensen JG, Li G (2003). In vivo antitumor activity of SU11248, a novel tyrosine kinase inhibitor targeting vascular endothelial growth factor and platelet-derived growth factor receptors: determination of a pharmacokinetic/pharmacodynamic relationship. Clin Cancer Res.

[10] Folkman J (2006). Antiangiogenesis in cancer therapy-endostatin and its mechanisms of action. Exp Cell Res.

[11] Xu HM, Yin R, Chen L, Siraj S, Huang X, Wang M (2008). An RGD-modified endostatin-derived synthetic peptide shows antitumor activity in vivo. Bioconjug Chem.

[12] Wickström SA, Alitalo K, Keski-Oja J (2004). An endostatin-derived peptide interacts with integrins and regulates actin cytoskeleton and migration of endothelial cells. J Biol Chem.

[13] Xu H, Pan L, Ren Y, Yang Y, Huang X, Liu Z (2011). RGD-modified angiogenesis inhibitor HM-3 dose: dual function during cancer treatment. Bioconjug Chem.

[14] Ridley AJ, Schwartz MA, Burridge K, Firtel RA, Ginsberg MH, Borisy G (2003). Cell migration: integrating signals from front to back. Science..

[15] Wickström SA, Alitalo K, Keski-Oja J (2003). Endostatin associates with lipid rafts and induces reorganization of the actin cytoskeleton via down-regulation of RhoA activity. J Biol Chem.

[16] Borges E, Jan Y, Ruoslahti E (2000). Platelet-derived growth factor receptor beta and vascular endothelial growth factor receptor 2 bind to the beta 3 integrin through its extracellular domain. J Biol Chem.

[17] Soldi R, Mitola S, Strasly M, Defilippi P, Tarone G, Bussolino F (1999). Role of alphavbeta3 integrin in the activation of vascular endothelial growth factor receptor-2. EMBO J.

[18] Simons K, Ikonen E (1997). Functional rafts in cell membranes. Nature..

[19] Anderson RG (1998). Thecaveolae membrane system. Annu Rev Biochem.

[20] Smart EJ, Graf GA, McNiven MA, Sessa WC, Engelman JA, Scherer PE (1999). Caveolins, liquid-ordered domains, and signal transduction. Mol Cell Biol.

[21] Mitra SK, Schlaepfer DD (2006). Integrin-regulated FAK-Src signaling in normal and cancer cells. Curr Opin Cell Biol.

[22] Huveneers S, Danen EHJ (1999). Adhesion signaling-crosstalk between integrins. Src and Rho J Cell Sci.

[23] Eliceiri BP (2001). Integrin and growth factor receptor crosstalk. Circ Res.

[24] Di Q, Cheng Z, Kim W, Liu Z, Song H, Li X (2013). Impaired cross-activation of β3 integrin and VEGFR-2 on endothelial progenitor cells with aging decreases angiogenesis in response to hypoxia. Int J Cardiol.

RETRACTED

[25] Mahabeleshwar GH, Feng W, Reddy K, Plow EF, Byzova TV (2007). Mechanisms of integrin-vascular endothelial growth factor receptor cross-activation in angiogenesis. Circ Res.

[26] Schoenwaelder SM, Burridge K (1999). Bidirectional signaling between the cytoskeleton and integrins. Curr Opin Cell Biol.

[27] Klinghoffer RA, Sachsenmaier C, Cooper JA, Soriano P (1999). Src family kinases are required for integrin but not PDGFR signal transduction. EMBO J.

[28] Smart EJ, Ying YS, Mineo C, Anderson RG (1995). A detergent-free method for purifying caveolae membrane from tissue culture cells. Proc Natl Acad Sci U S A.

[29] Olsson AK, Johansson I, Akerud H, Einarsson B, Christofferson R, Sasaki T (2004). The minimal active domain of endostatin is a heparin-binding motif that mediates inhibition of tumor vascularization. Cancer Res.

[30] Karumanchi SA, Jha V, Ramchandran R, Karihaloo A, Tsiokas L, Chan B (2001). Cell surface glypicans are low-affinity endostatin receptors. Mol Cell.

[31] Norton KA, Han Z, Popel AS, Pandey NB (2014). Antiangiogneic cancer drug sunitinib exhibits unexpected proangiogenic effects on endothelial cells. Onco Targets Ther.

[32] Shen H, Han H, Hu J, Zhang X, Wang J, Wang W (2014). PEGylated HM-3 presents anti-rheumatic bioactivity by inhibiting angiogenesis and inflammation. J Materials Chem B.

[33] Furuya K, Kaku Y, Yoshida K, Joh K, Kurosaka D (2014). Therapeutic effects of sunitinib, one of the anti-angiogenetic drugs, in a murine arthritis. Mod Rheumatol.

[34] Demali KA, Burridge K (2003). Coupling membrane protrusion and cell adhesion. J Cell Sci.

[35] Webb DJ, Parsons JT, Horwitz AF (2002). Adhesion assembly, disassembly and turnover in migrating cells – over and over and over again. Nat Cell Biol.

[36] Brugnera E, Haney L, Grimsley C, Lu M, Walk SF, Tosello-Trampont AC (2002). Unconventional Rac-GEF activity is mediated through the Dock180-ELMO complex. Nat Cell Biol.

[37] ten Klooster JP, Jaffer ZM, Chernoff J, Hordijk PL (2006). Targeting and activation of Rac1 are mediated by the exchange factor beta-pix. J Cell Biol.

[38] Arthur WT, Petch LA, Burridge K (2000). Integrin engagement suppresses RhoA activity via a c-Src-dependent mechanism. Curr Biol.

[39] Dubash AD, Wennerberg K, Garcia-Mata R, Menold MM, Arthur WT, Burridge K (2007). A novel role for Lsc/p115 RhoGEF and LARG in regulating RhoA activity downstream of adhesion to fibronectin. J Cell Sci.

[40] Lim Y, Lim ST, Tomar A, Gardel M, Bernard-Trifilo JA, Chen XL (2008). PyK2 and FAK connections to p190Rho guanine nucleotide exchange factor regulate RhoA activity, focal adhesion formation, and cell motility. J Cell Biol.

RETRACTED

[41] Yamada KM, Even-Ram S (2002). Integrin regulation of growth factor receptors. Nat Cell Biol.

[42] Burridge K, Wennerberg K (2004). Rho and Rac take center stage. Cell..

[43] Salanueva IJ, Cerezo A, Guadamillas MC, del Pozo MA (2007). Integrin regulation of caveolin function. J Cell Mol Med.

